This article has been retracted.

# The Efficacy of Minocycline Hydrochloride Combined with Multiple Antibiotic Paste in Elderly Patients with Chronic Periodontitis and Concomitant Pulp Lesions

**DOI:** 10.1155/2022/7604741

**Published:** 2022-07-04

**Authors:** Qiang Chen, Wen Yan, Nan Geng

**Affiliations:** ^1^Department of Periodontics, Suzhou Stomatological Hospital, Suzhou, Jiangsu 215000, China; ^2^Center of Stomatology, The Second Affiliated Hospital of Soochow University, No 1055 Sanxiang Road, Soochow 215004, China; ^3^Jiangsu Key Laboratory of Oral Diseases, Nanjing Medical University, Nanjing, Jiangsu 210029, China; ^4^Department of TeZhen, Affiliated Stomatological Hospital of Nanjing Medical University, Nanjing, Jiangsu 210029, China

## Abstract

**Objective:**

To explore the efficacy of Minocycline hydrochloride combined with multiple antibiotic pastes in the treatment of chronic periodontitis with concomitant pulp lesions in elderly patients, as well as to analyze the changes in the levels of inflammatory markers.

**Methods:**

100 patients suffering from chronic periodontitis with concomitant pulp lesions treated in our hospital from July 2018 to January 2020 were selected as the study subjects, and were randomly assigned to either an experimental group (*n* = 50) or a control group (*n* = 50). Patients in the experimental group were treated with Minocycline hydrochloride combined with multiple antibiotic pastes, while those in the control group were treated with Minocycline hydrochloride alone. The treatment efficacy in the two groups was then assessed using such factors as periodontal probing depth, dental plaque index, gingival index, periodontal attachment level, and the presence or absence of adverse effects. We also measured and compared the levels of inflammatory markers such as CRP, TNF-*α*, IL-1*β*, IL-5, IL-6, and others in both groups, before treatment, as well as after a week of treatment.

**Results:**

There was a statistically significant difference in the treatment efficacy between the two groups (*P* < 0.05), with a higher treatment efficacy seen in the experimental group as compared to the control group. When compared to the control group, the experimental group had lower depths of periodontal probing, lower dental plaque indices, lower gingival indices, lower periodontal attachment levels, as well a significantly lower incidence of adverse reactions (*P* < 0.05). Before treatment, the levels of inflammatory markers such as CRP, TNF-*α*, IL-1*β*, IL-5, and IL-6 were elevated in both groups. After a week of treatment, there were reductions in the levels of inflammatory markers in both groups, but a more significant reduction was seen in the experimental than in the control group (*P* < 0.05).

**Conclusion:**

Minocycline hydrochloride combined with various antibiotic pastes is more effective in the treatment of chronic periodontitis with concomitant pulp lesions in elderly patients than monotherapy with Minocycline hydrochloride alone.

## 1. Introduction

Chronic periodontitis is a common disease of the oral cavity among adults, consisting of chronic inflammation of the periodontal tissues that is caused by the accumulation of profuse amounts of dental plaque. It initially begins as gingivitis and then progresses into chronic periodontitis, which may be punctuated by periods of rapid progression (the so-called “bursts of destruction”). The etiology is complex and is caused by dental plaque, calculus, traumatic occlusion, and other factors including food impaction and poor restorations. Symptoms of the disease include redness or bleeding of the gums while brushing teeth, recurrent swelling of the gums, halitosis (bad breath), and loosening of the teeth [1–3]. However, symptoms are usually not apparent in the early stages of the disease, and in many individuals, the disease has progressed significantly before they seek medical attention. It is important to diagnose chronic periodontitis in its early stages to prevent severe and irreversible damage to the protective and supportive structures of the tooth. When the opportunity of treating the disease in its early stages is missed, the treatment options left are chiefly surgical, such as dental extraction among others. However, these forms of treatment are expensive, and a proportion of patients are not able to afford them [4–6]. Such patients are then condemned to long periods of pain, much to the detriment of their physical and mental health. Chronic periodontitis is usually complicated by the development of lesions in the dental pulp.

At present, the pharmacological treatment for chronic periodontitis is done using the drug Minocycline hydrochloride. Minocycline hydrochloride belongs to a class of drugs known as Tetracyclines that mainly work by reversibly binding to the 30 S subunit of the bacterial ribosome, thus preventing the addition of amino acids to growing peptides and effectively inhibiting protein synthesis. Common side effects of the drug include nausea, vomiting, diarrhea, a feeling of lightheadedness, and dizziness [7–9]. These are usually mild. However, rare but potentially serious side effects may occur and include intracranial hypertension (greater risk of this side effect for obese women of childbearing age, and it usually goes away when the drug is discontinued), and pseudomembranous colitis (also known as antibiotic-associated colitis). In addition, monotherapy using minocycline hydrochloride alone fails to achieve the desired outcome in some patients. Multiple antibiotic paste is a paste that is composed of equal amounts of multiple antibiotics, mainly ciprofloxacin, clindamycin, and metronidazole. It has considerable activity against a range of bacteria and achieves excellent control of bacterial infections. It is against this backdrop that this study now aims to evaluate and compare the treatment efficacy of minocycline hydrochloride combined with multiple antibiotic paste in treating chronic periodontitis, to that of using minocycline hydrochloride alone. The study subjects are patients suffering from chronic periodontitis with concomitant pulp lesions, assigned to either an experimental group or a control group. The treatment efficacy in the two groups will be assessed using such factors as depth of periodontal probe, dental plaque index, gingival index, periodontal attachment level, and the presence or absence of adverse effects. We shall also measure and compared the levels of inflammatory markers such as CRP, TNF-*α*, IL-1*β*, IL-5, IL-6, and others in both groups, before treatment, as well as after a week of treatment.

## 2. Materials and Methods

### 2.1. General Materials

100 patients with chronic periodontitis and concomitant pulp lesions treated in our hospital from July 2018 to January 2020 were selected as the study subjects, and were assigned to either the experimental group (*n* = 50) or to the control group (*n* = 50). and an experimental group(*n* = 50). Patients in the experimental group were aged between 55 and 79 years old, while those in the control group were aged between 55 and 81 years old.

### 2.2. Inclusion and Exclusion Criteria

Inclusion criteria: Patients that met the following criteria were included in the study:

① Patients with chronic periodontitis and concomitant pulp lesions.
② Patients aged at least 55 years old.
③ Patients without other organic diseases, coagulation disorders, and those that had not used any anticoagulants recently.
④ Patients without a history of drug allergy or drug abuse.

It is worth stating that approval from the ethics committee of our hospital, as well as informed consent by the study subjects, was duly obtained. Participation in the study was entirely voluntary.

Exclusion criteria: The following patients were excluded from the study:

① Patients who were recently hospitalized for treatment of cardio-cerebrovascular diseases such as myocardial infarction, cerebral infarction, cerebral hemorrhage, etc.
② Patients who had consciousness disorders, and could not cooperate with this study.
③ Patients who did not want to take part in the study, or whose relatives did not want them to take part in the study.

## 3. Methods

All patients underwent routine examination of the oral cavity, and corresponding treatment plans were developed. Patients in the control group were treated with Minocycline hydrochloride (manufactured by Wyeth Pharmaceutical Co. Ltd. National Medicine Zhunzi No. H10960010). The root canal was irrigated with a mixture of sodium chloride and hydrogen peroxide, rinsed, and then dried. The inside of the root canal was infused with Zinc oxide eugenol paste (manufactured by Shanghai Qingpu Dental Material Factory, batch number: National Food and Drug Administration (Test) No. 3060191). FC cotton dipped in 2% iodophenol was then placed on the inside of the root canal, sealing it after ensuring that there was no gap in the root canal [10–12]. Minocycline hydrochloride was then injected into the periodontal pocket. Patients were not allowed to gargle during treatment with Minocycline hydrochloride. For patients in the experimental group, the root canal was irrigated using a mixture of sodium chloride and hydrogen peroxide after opening the pulp cavity and expanding the root canal. They were then injected with minocycline hydrochloride and multiple antibiotic paste after the root canal had dried. The multiple antibiotic paste was composed of ciprofloxacin (manufactured by Jiangsu Chenpai Pharmaceutical Group Co. Ltd, National Medicine Zhunzi No. H32021943), clindamycin (manufactured by North China Pharmaceutical Co. Ltd, National Medicine Zhunzi No. H20070107), and metronidazole (manufactured by Huazhong Pharmaceutical Co. Ltd, National Pharmaceutical Zhunzi No. H42020404), in a ratio of 1 : 1 : 1. When the root canal was filled with the paste, it was then sealed with Zinc oxide eugenol. Minocycline hydrochloride was injected into the periodontal pocket, and, as was the case for the control group, patients were not allowed to gargle during treatment with minocycline hydrochloride.

### 3.1. Observation Indicators

Treatment efficacy in the two groups was assessed and compared, using such factors as periodontal probing depth (PD), dental plaque index (PLI), gingival index (GI), periodontal attachment level (AL), and the presence or absence of adverse reactions. Treatment was considered to be significantly effective if, after a week of treatment, there was more than 50% reduction in GI, more than 2 mm reduction in PD, and a significant reduction of inflammation and pulp lesions. It was considered effective if, after a week of treatment, there was no more than 50% reduction in GI and no more than 2 mm reduction in PD. Lastly, treatment was considered to be ineffective if, after a week of treatment, there was very little change in the inflammation and pulp lesions. X-rays were used to check the state of the patient's alveolar bone.

We also measured and compared the levels of inflammatory markers such as CRP, TNF-*α*, IL-1*β*, IL-5, IL-6, and others in both groups, before treatment, as well as after a week of treatment. 5 ml of fasting venous blood was collected, an anticoagulant was added, the serum was obtained after centrifugation, and the DG5031 enzyme-linked immunosorbent assay was produced by Shanghai Kehuai Instrument Co., Ltd. was used to detect CRP, TNF-*α*, IL-1*β*, IL-5, and IL-6 levels.

### 3.2. Statistical Processing

All the relevant materials and data in this study were processed and analyzed using the SPSS20.0 software. The measurement data was expressed as (±*s*) using the *t* test, while the enumeration data was expressed as [*n* (%)] using the *X*^2^ test. A *P* value of less than 0.05 (i.e., *P* < 0.05) is indicative of a statistically significant difference.

## 4. Results

### 4.1. Baseline Data

There was no significant statistical difference in the general data of the patients, such as gender, age, and length of disease course (*P* > 0.05). See Table 1 for illustration.

### 4.2. Comparison of Efficacy Rate

The efficacy rate is calculated as the total number of patients in whom treatment was either significantly effective or effective, expressed as a percentage of the total number of patients that were treated. Our results show that there was a significantly higher efficacy rate in the experimental group than in the control group (88% vs 60%, *P* < 0.05). See Table 2 for illustration.

### 4.3. Comparison of Periodontal Indices

After a week of treatment, we compared the PD, PLI, GI, and AL of patients in the two groups. The results showed that patients in the experimental group had significantly lower periodontal indices than those in the control group (*P* < 0.05), suggesting that treatment with Minocycline hydrochloride combined with multiple antibiotic paste helps in reducing periodontal indices during the treatment of elderly patients with chronic periodontitis and concomitant pulp lesions. See Figure 1 for illustration.

### 4.4. Comparison of the Incidence of Adverse Reactions

After a week of treatment, we compared the incidence of adverse reactions such as nausea, itching of the skin, and gingival swelling in patients from both groups. The results showed that adverse reactions did occur in patients from both groups, but the incidence was significantly lower in the experimental group than in the control group (6% vs 22%, *P* < 0.05), indicating that treatment with Minocycline hydrochloride combined with multiple antibiotic paste helps in reducing the incidence of adverse reactions that may occur during the treatment of elderly patients with chronic periodontitis and concomitant pulp lesions. See Table 3 for illustration.

### 4.5. Comparison of Inflammatory Markers

We measured and compared the levels of inflammatory markers such as CRP, TNF-*α*, IL-1*β*, IL-5, IL-6, and others in both groups, before treatment, as well as after a week of treatment. The results showed that there was a significant reduction in the levels of inflammatory markers in both groups after a week of treatment, as compared to before treatment (*P* < 0.05). However, more profound reductions were seen in the experimental group than in the control group (*P* < 0.05). See Figures 2 and 3 for illustration (see Figure 4.

## 5. Discussion

The results of this study show that treatment using Minocycline hydrochloride and multiple antibiotic paste was more effective than treatment using Minocycline hydrochloride alone. The treatment efficacy in the experimental group was higher than that in the control group (*P* < 0.05). Our results also show that after a week of treatment, greater reductions in PD, GI, PLI, AL, and pulp lesions were produced following treatment with minocycline hydrochloride and multiple antibiotic paste than with minocycline hydrochloride alone. Adverse reactions such as nausea, itching of the skin, and gingival swelling occurred in patients from both groups, but the incidence of said adverse reactions was significantly lower in the experimental group than in the control group (6% vs 22%, *P* < 0.05), indicating that treatment with Minocycline hydrochloride combined with multiple antibiotic paste helps in reducing the incidence of adverse reactions. In the same vein, a reduction in the levels of inflammatory markers was seen in both groups after a week of treatment (*P* < 0.05), but the reduction was more pronounced in the experimental group than in the control group (*P* < 0.05). The potential mechanism is that Minocycline hydrochloride has a significant anti-inflammatory effect and a broad antibacterial spectrum, can maintain a high local concentration for a long time, and exert a long-term antibacterial effect. It can accelerate the attachment of periodontal tissue by promoting the regeneration of fibroblasts. Repairing periodontal and pulpal joint lesions can not only play a long-term antibacterial effect in the treatment of chronic periodontitis but also have the effect of repairing and regenerating periodontal tissue. Moreover, the multi-antibiotic paste is prepared with metronidazole, clindamycin, and ciprofloxacin, which can not only effectively control anaerobic infection, but also maintain a stable drug concentration for a long time, which plays an important role in controlling recurrence. Keles Yucel et al. [13] proposed that IL-6 expression in patients with chronic periodontitis was significantly high at the onset of chronic periodontitis, and significantly reduced following treatment for one month, findings that are consistent with the findings of our study.

## 6. Conclusion

In conclusion, treatment of chronic periodontitis and concomitant pulp lesions in elderly patients using minocycline hydrochloride and multiple antibiotic paste produces higher efficacy rates than monotherapy using minocycline hydrochloride alone. It produces significant reductions in periodontal indices, inflammatory markers, and pulp lesions. It is an approach that is worthy of more widespread promotion and application.

## Figures and Tables

**Figure 1:** Comparison of periodontal indices. Note: the *X*-axis indicates the PD (mm), PLI, GI, and AL (mm) while the *Y*-axis represents the expression data of each periodontal index. The PD, PLI, GI, and AL of patients in the experimental group were (3.16 ± 0.75) mm, (0.84 ± 0.11), (1.44 ± 0.57), and (2.66 ± 1.00) mm, respectively. The PD, PLI, GI, and AL of patients in the control group were (4.38 ± 0.99) mm, (1.12 ± 0.35), (2.19 ± 0.73), and (3.87 ± 1.25) mm, respectively, ^*∗*^indicates the comparison of the PD (mm) between the experimental group and the control group (*t* = 6.95, *P* < 0.001)^*∗∗*^ indicates the comparison of the PLI between the experimental group and the control group (*t* = 5.40, *P* < 0.001) ^*∗∗∗*^ indicates the comparison of GI between the experimental group and the control group (*t* = 5.73, *P* < 0.001) ^*∗∗∗∗*^ indicates the comparison of AL (mm) between the experimental group and the control group (*t* = 5.34, *P* < 0.001).

**Figure 2:** Comparison of levels of inflammatory markers in the experimental group before and after treatment. The levels of CRP, TNF-*α*, IL-1*β*, IL-5, and IL-6 in the experimental group before treatment were (4.06 ± 1.23) *μ*g/L, (6.01 ± 2.15) ng/L, (8.00 ± 2.59) ng/L, (11.58 ± 3.41) *μ*/L, (ng/L), and (7.51 ± 3.01) ng/L, respectively. The levels of CRP, TNF-*α*, IL-1*β*, IL-5, and IL-6 in the experimental group after treatment were (1.64 ± 0.77) *μ*g/L, (3.19 ± 1.03) ng/L, (4.13 ± 1.91) ng/L, (6.99 ± 2.38) *μ*/L, and (3.05 ± 0.79) ng/L, respectively. A is a comparison of the CRP (*μ*g/L) level before and after treatment in the experimental group (*t* = 11.79, *P* < 0.001). B is a comparison of the TNF-*α* (ng/L) level in the experimental group before and after treatment (*t* = 8.36, *P* < 0.001). C is a comparison of the IL-1*β* (ng/L) level before and after treatment in the experimental group (*t* = 8.50, *P* < 0.001). D is a comparison of the IL-6 (ng/L) level before and after treatment in the experimental group (*t* = 10.13, *P* < 0.001). E is a comparison of the IL-5 (*μ*/L) level before and after treatment in the experimental group (*t* = 7.80, *P* < 0.001).

**Figure 3:** Comparison of levels of inflammatory markers after treatment. The levels of CRP, TNF-*α*, IL-1*β*, IL-5, and IL-6 in the experimental group were (1.64 ± 0.77) *μ*g/L, (3.19 ± 1.03) ng/L, (4.13 ± 1.91) ng/L, (6.99 ± 2.38) *μ*/L, and (3.05 ± 0.79) ng/L, respectively. The levels of CRP, TNF-*α*, IL-1*β*, IL-5, and IL-6 in the control group were (2.57 ± 1.06) *μ*g/L, (4.98 ± 2.14) ng/L, (6.00 ± 2.59) ng/L, (8.17 ± 3.14) *μ*/L, and (4.89 ± 1.97) ng/L, respectively. A is a comparison of the CRP (*μ*g/L) level between the two groups after a week of treatment (*t* = 5.02, *P* < 0.001). B is a comparison of the TNF-*α* (ng/L) level between the two groups after a week of treatment (*t* = 5.33, *P* < 0.001). C is a comparison of the IL-1*β* (ng/L) level between the two groups after a week of treatment (*t* = 4.11, *P* < 0.001). D is a comparison of the IL-6 (ng/L) level between the two groups after a week of treatment (*t* = 6.13, *P* < 0.001). E is a comparison of the IL-5 (*μ*/L) level between the two groups after a week of treatment (*t* = 2.12, *P*=0.04).

**Figure 4:** Comparison of levels of inflammatory markers in the control group before and after treatment. The levels of CRP, TNF-*α*, IL-1*β*, IL-5, and IL-6 in the control group before treatment were (4.30 ± 1.68) *μ*g/L, (6.39 ± 3.30) ng/L, (8.33 ± 3.96) ng/L, (11.93 ± 4.08) *μ*/L, and (7.96 ± 3.69) ng/L, respectively. The levels of CRP, TNF-*α*, IL-1*β*, IL-5, and IL-6 in the control group after a week of treatment were (2.57 ± 1.06) *μ*g/L, (4.98 ± 2.14) ng/L, (6.00 ± 2.59) ng/L, (8.17 ± 3.14) *μ*/L, and (4.89 ± 1.97) ng/L, respectively. A is a comparison of the CRP (*μ*g/L) level before and after treatment in the control group (*t* = 6.16, *P* < 0.001). B is a comparison of the TNF-*α* (ng/L) level before and after treatment in the control group (*t* = 2.53, *P*=0.01). C is a comparison of the IL-1*β* (ng/L) level before and after treatment in the control group (*t* = 3.48, *P* < 0.001). D is a comparison of the IL-6 (ng/L) levels before and after treatment in the control group (*t* = 5.19, *P* < 0.001). E is a comparison of the IL-5 (*μ*/L) level before and after treatment in the control group (*t* = 5.16, *P* < 0.001).

**Table 1:** Comparison of general data of the patients ($\bar{x}$ ± *s*).

Group	Experimental group	Control group	*t*/*X*^2^	*P*
Gender (male/female)	26/24	25/25	0.04	0.84
Age (years old)	68.34 ± 6.72	69.08 ± 6.52	0.56	0.58
Height (cm)	164.08 ± 10.30	163.77 ± 10.56	0.15	0.88
Weight (kg)	66.52 ± 11.05	65.71 ± 12.54	0.34	0.73
Course (months)	6.36 ± 2.15	7.09 ± 2.08	1.73	0.09
History of smoking (years)	13.75 ± 3.39	14.00 ± 3.34	0.37	0.71
History of drinking (years)	15.37 ± 2.37	15.07 ± 2.55	0.61	0.54
Hypertension (cases)	36	33	0.42	0.52
Diabetes (cases)	20	22	0.16	0.69
Hyperlipidemia (cases)	13	15	0.20	0.66

**Table 2:** Comparison of efficacy rate.

Group	Significantly effective	Effective	Ineffective	Total efficacy rate (%)
Experimental group	29	15	6	88%
Control group	8	22	20	60%
*X* ^2^				10.19
*P*				0.001

**Table 3:** Comparison of the incidence of adverse reactions.

Group	Nausea	Skin itching	Gingival swelling	Incidence of adverse reactions (%)
Experimental group	2	0	1	6%
Control group	6	2	3	22%
*X* ^2^				5.32
*P*				0.02

## Data Availability

No data were used to support this study.

## References

[1] (2020). Comparison of subgingival irrigation effect of boric acid 0.5% and povidone-iodine 0.1% on chronic periodontitis﻿ treatment. *Oral Health & Preventive Dentistry*.

[2] (2020). A retrospective study on the crestal bone loss associated with different implant surfaces in chronic periodontitis patients under maintenance. *Clinical Oral Implants Research*.

[3] Biewer B., Rompen E., Mittelbronn M., Quatresooz P., Kleine Borgmann F. (2020). Effects of minocycline hydrochloride on extra‐skeletal bone formation in a guided bone generation model. A comparative histomorphometric study in rat calvaria. *Clinical Oral Implants Research*.

[4] Cheah C. W., Al‐Maleki A. R., Vadivelu J. (2020). Salivary and serum cathelicidin LL‐37 levels in subjects with rheumatoid arthritis and chronic periodontitis. *International Journal of Rheumatic Diseases*.

[5] He S.-L., Hou H.-J., Wang J.-H. (2020). Determining the minimal important difference of the oral health impact profile for chronic periodontitis. *Journal of Clinical Periodontology*.

[6] Aral C. A., Ölçer S. N., Aral K., Kapila Y. (2020). Oxidative stress, neutrophil elastase and IGFBP7 levels in patients with oropharyngeal cancer and chronic periodontitis. *Oral Diseases*.

[7] El‐Makaky Y., Abdalla Hawwam S., Hifnawy T. (2020). Salivary tumor necrosis factor‐alpha to detect the severity of erectile dysfunction: a randomized clinical trial. *Oral Diseases*.

[8] Gao H., Xu J., Lu H., Meng H., Hou J. (2020). Calprotectin levels in gingival crevicular fluid and serum of patients with chronic periodontitis and type 2 diabetes mellitus before and after initial periodontal therapy. *Journal of Periodontal Research*.

[9] Saiki K., Urano-Tashiro Y., Takahashi Y. (2020). Reassessment of minimal media reveals differences in growth among porphyromonas gingivalis standard strains. *Journal of Oral Biosciences*.

[10] Sun Y., Zhao B., Li Z., Wei J. (2020). Beneficial effects of glycyrrhizin in chronic periodontitis through the inhibition of inflammatory response. *Dose-Response*.

[11] Howard R., Zubko O., Bradley R. (2020). Minocycline at 2 different dosages vs placebo for patients with mild alzheimer disease: a randomized clinical trial. *JAMA Neurology*.

[12] Vohra F., Bukhari I. A., Sheikh S. A., Albaijan R., Naseem M., Hussain M. (2020). Effectiveness of scaling and root planing with and without adjunct probiotic therapy in the treatment of chronic periodontitis among *shamma* users and non‐users: a randomized controlled trial. *Journal of Periodontology*.

[13] Keles Yucel Z. P., Keles G. C., Avci B., Cetinkaya B. O. (2020). Nonsurgical periodontal therapy reduces salivary and gingival crevicular fluid YKL-40 and IL-6 levels in chronic periodontitis. *Oral Health & Preventive Dentistry*.

